# Hierarchical Attention-Based Multimodal Fusion Network for Video Emotion Recognition

**DOI:** 10.1155/2021/5585041

**Published:** 2021-09-25

**Authors:** Xiaodong Liu, Songyang Li, Miao Wang

**Affiliations:** School of Computing Henan University of Engineering, Zhengzhou, China

## Abstract

The context, such as scenes and objects, plays an important role in video emotion recognition. The emotion recognition accuracy can be further improved when the context information is incorporated. Although previous research has considered the context information, the emotional clues contained in different images may be different, which is often ignored. To address the problem of emotion difference between different modes and different images, this paper proposes a hierarchical attention-based multimodal fusion network for video emotion recognition, which consists of a multimodal feature extraction module and a multimodal feature fusion module. The multimodal feature extraction module has three subnetworks used to extract features of facial, scene, and global images. Each subnetwork consists of two branches, where the first branch extracts the features of different modes, and the other branch generates the emotion score for each image. Features and emotion scores of all images in a modal are aggregated to generate the emotion feature of the modal. The other module takes multimodal features as input and generates the emotion score for each modal. Finally, features and emotion scores of multiple modes are aggregated, and the final emotion representation of the video will be produced. Experimental results show that our proposed method is effective on the emotion recognition dataset.

## 1. Introduction

Emotion recognition is an important content of a comprehensive understanding of video scenes. It can help us understand humans emotions shown in a video clip. Particularly, understanding such emotions has a wide range of applications [1]. For example, video recommendation services can find users' interests and recommend the corresponding videos to them based on obtained video emotion. The emotion recognition platform can be used to recognize the potential suspicious person on intelligent security. Thus, recognition of the emotional states of humans from videos has been attracting more and more attention in recent years.

Previous research on video emotion recognition has mainly focused on exploring facial features. The facial action coding system (FACS) [2] encodes facial expression through facial movement in action units. It is extracted from face images and belongs to low-level features. Recently, with the success of deep convolution neural networks (CNNs) in the field of image classification and object detection, researchers attempt to extract face features based on deep neural networks to further improve the performance of emotion recognition [3, 4]. However, it cannot model the temporal evolution of emotion expression. Some researches model spatial and temporal clues of faces by 3D convolutional neural networks (C3D) and recurrent neural network (RNN) [5]. Some emotion recognition efforts have also been using body pose and audio features [6]. However, the context information is usually ignored in the previous research. Some studies have shown the importance of context in emotion recognition [7]. The emotion recognition accuracy can be further improved when the context information is incorporated.

Psychological researches [8] have been shown that context information can also provide important clues for emotion perception. Experiments in [9] show that recognition accuracy is improved when using both body and context information. Cheng [10] first extracts event, object, and scene features based on CNNs, and these features serve as context information and are further integrated by a context fusion network to generate a uniﬁed representation. However, these features are integrated by max/average pooling, and the difference of features in different video frames is not considered. Although the research of video emotion recognition has made great progress, it still has two major challenges.

1. *Scene Complexity*. Because of the complexity of the scene in the video, such as the difference of angle and distance of cameras, there will be a difference in pose and sharpness of humans in the video, which will lead to the difference of emotion discrimination. As an example, take a look at the images in Figure 1. Let us try to estimate what they feel. In Figure 1(a), emotional discrimination is different because of the different perspectives of the two images. It is easy to recognize that the emotion category of the right image is anger, and it is difficult to recognize the emotion category of the left image. In Figure 1(b), the angle of the two images is similar. However, due to the differences in sharpness, the right image can get more emotional cues than the left image. Similar to the human face, there are also emotional differences between contextual information (as is shown in Figure 2). Therefore, how to make full use of the emotional clues of different images is a significant challenge for video emotion recognition.
2. *Differences in Emotional Expressions of Different Modes in the Video*. Different modes contain different amounts of emotional information in different videos. For example, some videos contain more human images and fewer context images. Meanwhile, the face of the human has a rich emotional expression, such as the image sequences in Figure 2(e), so the emotion category through the facial emotion expression of humans can be easily recognized. In this case, we mainly use facial expression to recognize the emotion category of video, while context information is only used as a few emotional assistant clues. There are also some videos expressing rich emotion clues by scenes, and humans in videos contain fewer emotion clues, such as the image sequences in Figure 2(d). For this kind of video, the video emotion category can be mainly recognized by scenes. Therefore, in video emotional feature representation based on multimodal feature fusion, how to effectively solve the differences of different modal emotional expressions in the video is a significant challenge for video emotion recognition.

This paper addresses the problem of video emotion recognition considering the emotion difference between different modes and different images. The first contribution of our work is a multimodal human emotion dataset (MHED), which is described in Section 3. The MHED dataset is composed of short videos with a human, annotated with the emotional states defined by the psychologists Ekman and Friesen [11].

Using the MHED dataset, a hierarchical attention-based multimodal fusion network (HAMF) for video emotion recognition is trained, which is inspired by the quality-aware network [12] and attention cluster [13]. HAMF takes the image sequence of face, scene, and context as input and can learn a discrimination video emotion representation that can make full use of the differences of different modes and images. It consists of two attention-based modules.

*Multimodal Feature Extraction Module*. It has three CNN subnetworks, and each subnetwork consists of two branches. The first branch of the three CNN subnetworks takes the face, scene, and global images as input for extracting face features, scene features, and global context features. The other branch of the three subnetwork takes the middle representation of the face, scene, and global context features as input and generates an emotion score for each image. This branch is called a local attention network because it is used to generate the emotion score for each image of a modal approach. This is for the purpose of distinguishing global attention networks.

*Multimodal Feature Fusion Module*. Features of each modal are fed to the global attention network, which is used to generate emotion scores for different modes. The scores and features of multiple modes will be aggregated, and the final emotional representation of the video will be produced. Then, the final emotion representation of the video passes through a tiny fully connected network and is supervised by a softmax loss.

The main contributions of the paper are summarized as follows. Firstly, we constructed an MHED dataset, which mainly focuses on multimodal fusion for video emotion recognition in the wild. Secondly, the local attention network solves the problem of emotion difference of video frames, and the global attention network solves the problem of emotion difference of different modes.

The remainder of this paper is organized as follows. In Section 2, related work on video emotion recognition is discussed. Section 3 describes the MHED dataset.  Section 4 introduces the proposed hierarchical attention-based multimodal fusion network.  Section 5 gives experimental results.  Section 6 concludes the paper and gives our future work.

## 2. Related Work

### 2.1. Context-Aware Video Emotion Recognition

Most recent emotion recognition methods focus on exploring facial features based on deep neural networks [14]. In psychological researches [8], evidence and experiments show that contextual information such as pose and surrounding environment can also provide important clues for emotion recognition. Experiments in [9] show that when using both context and body information, the performance of emotion recognition outperforms that of using only body image or only context image. Yu-Gang Jiang [10] fuses rich context clues such as events, objects, and scenes to improve emotion recognition performance. Papers [9, 10] first extract high-level semantic features of facial and rich context clues, as inputs for a fusion network to derive a unified representation targeting the understanding of emotions. However, the relationship between facial and context is not considered. CACA-RNN [15] consists of two RNNs in a cascaded architecture, which processes both context and facial information to perform video emotion classification. In CACA-RNN, the relationship between face and its context is learned. In paper [5], to identify and exploit possible relationships among static facial features, motion features of humans, and temporal evolution of the audio features, a fusion network is proposed that merges cues from the different modes in one representation. Hoang et al. [16] proposed the emotional state prediction method based on visual relationship detection between the main target and the adjacent objects from the background to fully exploit the essences of context.

### 2.2. Multimodal Video Emotion Recognition

Multimodality image fusion can not only enhance visibility to human eyes but also mutually complement the limitations of each image. Zhu et al. [17] proposed an image fusion scheme based on image cartoon-texture decomposition and sparse representation, which can preserve the structure information and perform the detailed information of source images. Wang et al. [18] proposed a CNN-based medical image fusion algorithm to obtain a fused image with high visual quality and clear structure details. It fuses the pixel activity information of source images to realize the generation of weight maps. Vielzeuf et al. [19] proposed a multimodal fusion method, which combines VGG and C3d models as image feature extractor and explores the different temporal fusion network.

### 2.3. Attention-Based Video Emotion Recognition

Because the sparsity of emotion expression in video and human emotion can only be recognized in some specific moments during a long utterance, attention mechanism is used to aware of which time-frequency region of speech spectrogram is more emotion-relevant in the paper [20]. Lee et al. [21] learn spatiotemporal attention that selectively focuses on emotion salient parts within face videos. Barros et al. [22] propose a deep architecture that implements convolutional neural networks to learn the location of emotional expressions in a cluttered scene. Papers [20–22] use attention mechanisms selectively focusing on emotional salient parts. These papers only consider spatial attention mechanisms. There are also some researches that focus on spatial and temporal attention mechanisms. Temporal attention and band attention on multilayer LSTM are combined in the paper [23]. Band attention applies different levels of attention to different frequency bands of EEG signals, and temporal attention is used to determine where to analyze the next signal in order to suppress the redundant information. Huang et al. [24] propose a convolutional attention mechanism to learn the utterance structure relevant to the task for speech emotion recognition. Fan and Yunjie [25] can learn the weights of different model predictions so that the fusion of multimodal would make sense. Attention mechanisms that have been studied mainly study frame relationships or regions of interest of emotion. Zhang and Xu [26] adopt the sparse representation method to construct kernel functions, used to convert CNN features into kernelized features. It applies the sparse representation method to reduce the impact of noise contained in videos. Xu et al. [27] conduct concept selection to investigate the relations between high-level concept features and emotions. The discriminative concepts play important roles in emotion recognition. In this paper, different images of modal and different modes are assigned an emotion score, and this score represents the importance of images or modes.

## 3. MHED

The MHED dataset is constructed from videos that we manually downloaded from the Web, which mainly focuses on human emotion in the video. Six emotion categories are considered according to the well-known psychologists Ekman and Friesen [11], including “anger”, “disgust”, “fear”, “joy”, “sadness”, and “surprise”. The dataset contains a total number of 1066 videos, and each video has an annotated human. The video number is 638 for training, and the test video number is 428. There is no overlap between the training set and the test set. Figure 2 shows example frames of each emotion category from the MHED dataset. As shown in Figure 2, different images of the same video contain different amounts of emotional information. Meanwhile, the different modes also contain different amounts of emotional information. For example, in Figure 2(d), the scene contains abundant emotional clues, and it is easy to recognize that the emotion category is sadness. However, it is difficult to recognize the emotion category of Figure 2(f) from the scene of the video.

### 3.1. Dataset Annotation

The MHED dataset was manually annotated by 16 annotators.  Table 1 shows the gender and age distribution of annotators. As is shown in Table 1, these 16 annotators come from different age groups. The annotators cover the age range from 20 to 60, and each age group contains the same number of humans. Of the 16 annotators, 8 were male and 8 were female, and they are averagely distributed among all age groups.

In order to ensure the quality of the annotations, annotators first need to learn the definition of the emotional categories, given by psychologists Ekman and Friesen. Secondly, some video clips with emotion labels coming from the existing video emotion recognition dataset are exercised by annotators. After learning and practicing, annotators are asked to annotate our MHED dataset. In the case of emotion categories, we show a video clip and ask the annotators to select an emotion category that applies to that video. Each annotator independently annotates emotions, and the emotion catalog of a video marked by the most annotators is selected as the emotion label of the video. Furthermore, annotators also annotated the gender and age of humans in the video.

### 3.2. Database Statistics

Of the 1066 annotated videos, 37.15% are males and 62.85% are females. Their ages are distributed as follows: 5.9% children, 6.47% teenagers, and 87.63% adults. The dataset has a minimum number of 137 videos per category and an average duration of 15.76 seconds.  Table 2 summarizes more details.

## 4. Hierarchical Attention-Based Multimodal Fusion Network

In this section, the hierarchical attention-based multimodal fusion network (HAMF) will be described in detail. Specifically, our proposed framework is first introduced. Then, the local attention mechanism to extract the emotional score of each image is given. Finally, the multimodal fusion method based on the global attention mechanism is described.

### 4.1. Hierarchical Attention-Based Multimodal Fusion Network Framework

Context information including scene, body, pose, and surrounding environment can also provide different emotional pieces of information, which can help to improve the accuracy of emotion recognition. However, as discussed in Section 1, there is an obvious problem in the fusion of different images and different modes. To tackle this issue, a hierarchical attention-based multimodal fusion network as shown in Figure 3 is proposed, to enable us to model the fusion of different images and modes.

Speciﬁcally, our proposed HAMF network fuses multimodal features of a video to recognize video emotion. HAMF consists of two attention-based modules. The first module is a multimodal feature extraction module for generating emotion features of each modal. It has three CNN subnetworks, and each subnetwork consists of two branches. The first branch of the first CNN network takes images as input and extracts scene features for providing surrounding environment support. The first branch of the second CNN network takes images of the face as input and extracts face features for providing human feeling. The first branch of the third CNN network takes global images as input and extracts global context features, such as body and pose, for providing contextual support. The scene CNN and image CNN use the same input, but they use different networks and generate different features. The other branch of the three subnetworks takes the middle representation of the face, scene, and global features as input and generates an emotion score for each image. This branch is called a local attention network because it is used to generate the emotion score for each image of a modal approach. This is for the purpose of distinguishing global attention network which is used to generate emotion scores for different modes. Then, the emotion scores and image features of each modal will be aggregated, and the feature of each modal is produced. The other module is a multimodal feature fusion module for fusing multimodal features and generating the emotional representation of the video. Each modal's features pass through a global attention network and generate an emotion score for each modal. The features of multiple modes and their emotion scores will be aggregated, and the final emotion representation of the video will be produced. It will pass through a tiny fully connected network and is supervised by softmax loss.

The local attention network and the global attention network are trained separately. A training sample includes three video frame sequences: *s*_*a*_ is anchor, positive sample sequence *s*_*p*_ where its emotion is consistent with *s*_*a*_, and negative sample sequence *s*_*n*_ where its emotion is different from *s*_*a*_. Three video frame sequences propagate forward through the same CNN network and output the corresponding features *R*(*s*_*a*_), *R*(*s*_*p*_), *R*(*s*_*n*_). A set's representation *R*(*s*_*a*_) is supervised by triplet loss [28] *L*_*t*_, which is formulated as

(1) $$\begin{array}{c} {\text{L}}_{t}={\left\|R\left(s_{a}\right)-R\left(s_{p}\right)\right\|}^{2}-{\left\|R\left(s_{a}\right)-R\left(s_{n}\right)\right\|}^{2}+\delta , \end{array}$$

where *δ* is a very small positive number.

### 4.2. Multimodal Feature Extraction

Multimodal feature extraction module is used to extract face, scene, and global image features by three parallel CNN networks. Given an image sequence *S* of video V, faces are first extracted by faster-R-CNN [29] trained on the WIDER dataset [30], and the detected faces are resized to 224 × 224. Let *n* be the number of faces of the video V, and face sequences can be expressed as *F*={*f*_1_, *f*_2_,…, *f*_*n*_}. For convenience, in the experimental stage, we also selected *n* images from image sequences. Therefore, image sequences can be expressed as *S*={*I*_1_, *I*_2_,…, *I*_*n*_}. The features of each modal are extracted by an independent CNN network. VGG-face model [31] which is trained on the VGG-face dataset [31] as initialization is used to extract face features. It takes face images as input and generates face features. Scene features are extracted by VGG which is pretrained on the Places365 dataset [32]. It takes image sequences as input and generates scene features. The third CNN network takes the entire image as input and extracts global features for providing body, pose, and surrounding contextual information. Each of the three CNN networks consists of two branches, where the first branch extracts image features and the other branch generates emotion scores. It is split into two branches on the layer pool5. The first branch passes through a tiny fully connected network and is supervised by softmax loss, which optimizes the probability of each image. The second branch is an emotion score generation network, which is used to generate an emotion score. It can be expressed by a convolution layer and a fully connected layer that has only one cell (*L*1):

(2) $$\begin{array}{c} S_{i}=W_{0}^{L}\sigma \left(W_{{}_{1}}^{L}\times M_{i}+b_{1}\right)+b_{0}, \end{array}$$

where *S*_*i*_ denotes the emotion score of the *i*th modal, *M*_*i*_ is the middle representation of a feature of the *i*th modal, and *W*_0_^*L*^, *W*_1_^*L*^, *b*_1_, and *b*_2_ are parameters which can be learned through training. *σ*() is an active function. Here, we choose the rectified linear function for *σ*(). Similarly, we can also use two or three successive convolution layers and one fully connected layer that has only one cell, annotated by *L*2 and *L*3, respectively:

(3) $$\begin{array}{c} S_{i}=W_{0}^{L}\left(W_{2}^{L}\sigma \left(W_{{}_{1}}^{L}\times M_{i}+b_{1}\right)+b_{2}\right)+b_{0},\\ S_{i}=W_{0}^{L}\sigma \left(W_{3}^{L}\sigma W_{2}^{L}\sigma \left(W_{{}_{1}}^{L}\times M_{i}+b_{1}\right)+b_{2}+b_{3}\right)+b_{0}, \end{array}$$

where *W*_0_^*L*^, *W*_1_^*L*^, *W*_2_^*L*^, *W*_3_^*L*^, *b*_0_, *b*_1_, *b*_2_, and *b*_3_ are parameters which can be learned through training. In the experiments, the effect of the above different weighting functions will be compared.

Then, the fc6 layer emotion features and scores of all images are extracted. We use *X*_*i*_={*x*_*ij*_*|j*=1,2,…, *n*}which denotes the fc6 features of the *i*th modal and *S*_*i*_={*s*_*ij*_*|j*=1,2,…, *n*} which denotes the emotion scores of the *i*th modal. The final emotion representation of the *i*th modal is a linear combination of emotion features and its emotion score.

(4) $$\begin{array}{c} F_{i}=\sum_{j=1}^{n}x_{ij}\times s_{ij}. \end{array}$$

The final emotion representation is supervised by triplet loss [28], which minimizes variances of intraclass samples.

### 4.3. Multimodal Feature Fusion

The different modes can be efficiently combined to improve emotion recognition performance. The contribution of each modal is different in different videos. Thus, a global attention mechanism is used to combine these modes according to their contribution. Its responsibility is to evaluate the importance of each modal and then assign an emotion score for each modal. Multimodal features and their emotion scores will be aggregated together, and the final emotion representation of the video is produced.

Let *m* be the number of modes, and let *X*_*i*_ be the features of the *i*th modal. This paper uses three modes: face, scene, and global feature, and *X*_*i*_ is a 4096-dimensional vector, which is got by aggregating the fc6 feature and emotion score of all images of the *i*th modal. We can use a matrix *X* to represent a feature set containing *m* modes:

(5) $$\begin{array}{c} X=\left\{X_{1},X_{2},\ldots ,X_{m}\right\}. \end{array}$$

It should be noted here that the modes are unordered, and permuting the rows of the matrix cannot affect the results. The global attention results can essentially be expressed by

(6) $$\begin{array}{c} G\left(X\right)=\left(\alpha_{1}X_{1},\alpha_{2}X_{2},\ldots ,\alpha_{n}X_{m}\right), \end{array}$$

where *α*_*i*_ is the weight of the *i*th modal. It can be acquired through learning a linear mapping *W*_*i*_^*g*^ and can use a single fully connected layer that has only one cell (*G*1):

(7) $$\begin{array}{c} \alpha_{i}=W_{i}^{g}X_{i}+b, \end{array}$$

where *W*_*i*_^*g*^ and *b* are parameters which can be learned through training with standard backpropagation.

*Algorithms*. Similarly, we can also use two or three successive fully connected layers, annotated by *G*2 and *G*3, respectively:

(8) $$\begin{array}{c} \alpha_{i}=W_{i2}^{g}\sigma \left(W_{i1}^{g}X_{i}+b_{1}\right)+b_{2},\\ \alpha_{i}=W_{i3}^{g}\sigma \left(W_{i2}^{g}\sigma \left(W_{i1}^{g}X_{i}+b_{1}\right)+b_{2}\right)+b_{3}, \end{array}$$

where *W*_*i*1_^*g*^, *W*_*i*2_^*g*^, *b*_1_, and *b*_2_ are parameters which can be learned through training, and *σ*() is an active function. In the experiments, the effect of the above different weighting functions will be compared.

The multimodal features and their emotion scores generated by the global attention network are aggregated and generate a unified representation *F*:

(9) $$\begin{array}{c} F=\text{XG}{\left(X\right)}^{T}, \end{array}$$

where *X* is a feature set containing *m* modes and *G*(•) is used to generate emotion scores, which is described in formula (6). Then, the emotion representation F passed through two fully connected layers and is supervised by softmax loss.

## 5. Experiments

Our implementation is based on PyTorch deep learning framework. In our framework, the local attention network and the global attention network are trained separately. The learning rate is initialized as 0.001 and decreases to 10% every 6000 iterations. The whole training procedure stops at 25, 000 iterations. The momentum is set to 0.9. We uniformly partition an input video into 24 segments, in which one frame is randomly sampled to obtain 24 frames for one video.

### 5.1. Effect of Weighting Function

In this subsection, the effect of the weighting function of HAMF on emotion recognition performance is evaluated. First of all, the results of the local attention network are given. Three different weight functions of attention network *L*1, *L*2, and *L*3 as described in Section 4.2 are considered.  Table 3 gives the accuracy of emotion recognition of different modes by local attention network using different weighting functions. As shown in Table 3, on our MHED dataset, the accuracy of emotion recognition is different using different weighting functions in the local attention network. The weighting function *L*2 is slightly better than *L*1 and *L*1 is slightly better than *L*3 for face features and scene features. The weighting function *L*1 is slightly better than *L*2 and *L*3 for global features. We rely on the *L*2 weighting function for face and scene features and the *L*1 weighting function for global features as the default in all subsequent experiments. Secondly, the results of the global attention network are given. Three different weight functions of attention network *G*1, *G*2, and *G*3 as described in Section 4.3 are considered.  Table 4 gives the accuracy of emotion recognition by global attention network using different weighting functions. As shown in Table 4, on our MHED dataset, the accuracy of emotion recognition is different using different weighting functions in the global attention network. We can see that *G*2 is slightly better than *G*1 and *G*1 is slightly better than *G*3 for the global attention network. To further verify the effect of weight function, we conduct experiments on Ekman-6 [33] and VideoEmotion-8 [34] datasets, which will be described in detail in Section 5.5.  Table 5 gives the accuracy of emotion recognition of different modes by local attention network using different weighting functions on Ekman and VideoEmotion-8 datasets.  Table 6 gives the accuracy of emotion recognition by global attention network using different weighting functions on Ekman and VideoEmotion-8 datasets. These experiments show that a deeper attention network can get better results but when the number of layers of the attention network exceeds a certain degree, the accuracy will be degraded. This may stem from the expressive power of the attention network saturating as the size increases.

### 5.2. The Evaluation of Attention Mechanism

In this subsection, the performance of the local attention mechanism and global attention mechanism is evaluated. In order to validate the effectiveness of our local attention mechanism and global attention mechanism, we compare the following two average fusion approaches.

*Images Average Fusion (IAF)*. Image features of the face, scene, and context are extracted separately by three CNN networks without an attention mechanism. Then, these image features of each modal are aggregated by average pooling, and emotion features of the face modal, scene modal, and global modal of the video are obtained.

*Multimodal Fusion (MF).* The fc6 layer features of face modal, scene modal, and global modal are first extracted. Then, these features are fused by the concatenation method which is described in the paper [35]. These fused features are used as the input of a tiny fully connected network, which is supervised by the softmax loss function.

Firstly, the local attention mechanism is evaluated. In this experiment, the global attention network does not use the attention mechanism, and the local attention network uses and does not use attention mechanisms, respectively.  Table 7 gives the results of emotion recognition with local attention mechanism and without attention mechanism. As shown in Table 7, on our MHED dataset, the top-1 accuracy of local attention mechanism increases by 6.07%, 0.93%, and 2.11%, respectively, compared with the IAF method of face modal, scene modal, and context modal. We notice that the degree of improvement is different in different modals. The improvement of the face modal is much more than the scene modal. This is because emotion differences among different video frames are greater in the face modal. Secondly, the performance of the global attention mechanism is evaluated. The local attention network does not use attention mechanisms. The global attention network takes different modal features as input separately and generates an emotion score for each modal. The different modal features are fused according to their emotion score, and the final emotion representation of the video is produced.  Table 7 also gives the result of emotion recognition accuracy of MF and our global attention-based multimodal feature fusion network. As shown in Table 7, on our MHED dataset, the global attention mechanism increases the top-1 accuracy by 3.03% compared with the MF method without the global attention mechanism. Based on these two experiments, local attention mechanisms and global attention mechanisms outperform average fusion without attention mechanisms.

Table 7 also shows the comparison results of single mode and multimode. Our multimode method achieves 60.05% and 60.08% on no attention network and attention network, respectively, outperforming single-mode methods by clear margins. This is because multimode clues characterize the video from multiple perspectives.

### 5.3. Visualization of Hierarchical Attention Mechanism

In order to visualize the hierarchical attention mechanism, some image sequences in the test set and their corresponding emotional scores are shown in Figure 4. Figures 4(a) and 4(b) show facial sequences and their corresponding emotional scores. As shown in Figures 4(a) and 4(b), the emotional scores of different facial images of the same person are different because of the difference in their posture and angle. Some faces contain rich emotional cues, such as the second and third facial images in Figure 4(a), through which one can easily judge a person's emotions. Thus, HAMF gives these faces higher emotional scores. Some faces express fewer emotional cues, such as the 6th image in Figure 4(b), and they get lower emotional scores. Figures 4(c) and 4(d) show some image sequences and their corresponding scene emotional scores. The scene of images also contains certain emotional clues. In Figure 4(c), the difference of contained scene emotional cues in image sequence is little, so the emotional scores of these images have little difference. In Figure 4(d), the scene of the image sequence contains different emotional cues. The scene contains rich emotional cues in some images, such as the 7th and 8th images in Figure 4(d), which will be assigned higher emotional scores. Meanwhile, the scene contains few emotional cues in some images, such as the 4th image in Figure 4(d), which will get lower emotional scores. Similarly, as shown in Figures 4(e) and 4(f), there are also differences in emotional cues contained in global images; thus, they obtain different emotional scores.

Figure 5 shows the emotional scores of different modes of the image sequences in Figure 4. The number shown in the figure is the emotional score of each video obtained by the global attention network. For each video, the sum of the scores for the three modes is equal to 1. As shown in Figure 5, facial, scene, and context modes contain different emotional cues in different videos, so the emotional scores obtained by these three modes are different. For example, in Figures 5(a) and 5(b), the facial modality of videos contains the most amount of emotional information, so the facial modality has the highest emotional score. However, in Figure 5(c), the facial modality obtained a very low emotional score. Based on Figures 4 and 5, we can see that HAMF can make full use of the emotional differences between different images and modes to enhance discrimination of emotion recognition.

### 5.4. Comparison with State-of-the-Art Approaches

In this subsection, we compare the state-of-the-art performance in recent literature. To validate the effectiveness of our HAMF method, we compare the following state-of-the-art approaches.

*Quality-Aware Network (QAN)* [12]. It is mainly used to solve the quality difference between images. Image sequences of a video are sent to QAN, and features and scores of each image are generated. Then, features are integrated and the final feature of the video is produced.

*Attention Clusters* [13]. The fc6 layer features of all images of face modal, scene modal, and context modal are extracted. Then, they are sent to an attention network that uses a single fully connected layer that has only one cell. Features of each modal are concatenated according to the output of the attention network, and the emotion feature of each modal is produced. Finally, features of the three modes are concatenated and passed a fully connected layer and are supervised by softmax loss.

*Emotion Recognition in Context (ERC)* [9]. ERC consists of two main modules. Its first module takes the region of the image comprising the person and extracts the emotional feelings of the person, and the second module takes the entire image as input and extracts global features for providing the necessary contextual support. Then, these two features are fused by a fusion network. Finally, fusion features are integrated by the average pooling.

*Emotion in Context (EC)* [10]. Images' fc6 features of the event, object, and scene are extracted and integrated according to the average method. Then, three features are fused by a context fusion network.

*Temporal Multimodal Fusion (TMF)* [19]. Face feature is generated by vgg-lstm and c3d-lstm, and they are fused by the weight mean fusion method.

Table 8 shows the accuracy comparison of the above methods on the MHED dataset. As shown in Table 8, our hierarchical attention-based multimodal fusion network achieves a 3.27% top-1 performance gain on our MHED. The accuracy of QAN which only takes images as input is the lowest. The performance of multimodal feature fusion literature [9, 10] and spatial-temporal feature fusion network [22] are all better than QAN. This is because that QAN network only uses a single modal. Multimodal feature fusion network, which uses multiple modes, can achieve better performance. By the attention mechanism, the performance of the attention cluster [13] takes the fc6 features of the face, scene, and global images as inputs which are better than those feature fusion methods without an attention mechanism. Note that our work attains superior performance for two reasons: firstly, the local attention mechanism can distinguish the emotional differences of different images and can make full use of the emotional features of different images. Secondly, the global attention mechanism can distinguish the emotional differences of different modes and can make full use of the emotional features of different modes.

### 5.5. Result on Ekman-6 and VideoEmotion-8

In this section, we conduct experiments on Ekman-6 [33] and VideoEmotion-8 [34] datasets to further evaluate the effectiveness of our method.

The ekman-6 dataset contains 1637 videos, and it uses a training set of 819 videos and a testing set of 818 videos. There is no overlap between the training set and the test set. It was manually annotated by 10 annotators according to Ekman's theory [11] on six basic human emotion categories, with a minimum of 221 videos per category.

The videoEmotion-8 dataset contains 1101 videos collected from YouTube and Flickr. The average duration of videos is 107 seconds. It uses a training set of 734 videos and a testing set of 367 videos. There is no overlap between the training set and the test set. The experiments were conducted 10 times according to train/test splits provided by [34].

Table 9 gives top-1 accuracy (%) of different methods on Ekman-6 and VideoEmotion-8 datasets. As shown in Table 9, our context-aware attention fusion network achieves 2.69% and 1.36% performance gain on Ekman-6 and VideoEmotion-8 datasets, respectively. The accuracy of emotion in context [10] which has only fusion context information is the lowest. Xu et al. [33] studied the problem of transferring knowledge from heterogeneous external sources that can further improve accuracy. Kernelized feature [26] and concept selection [27] studied frame relationships or regions of interest of emotion, which further improve the accuracy. Graph-based network [36] utilizes the semantic relationships of different regions based on the graph convolutional network to improve accuracy. Our previous work CAAN [37] only solves the difference of contained emotion information in different images. The results show that our methods achieve state-of-the-art results on both Ekman-6 and VideoEmotion-8 datasets. This is because our method addresses the problem of emotion difference between different modes and images.

## 6. Conclusions

In this paper, we first build a dataset for human emotion recognition in video, named multimodal human emotion dataset (MHED). With the MHED dataset, a hierarchical attention-based multimodal fusion network (HAMF) for human emotion recognition in video is trained. HAMF uses a hierarchical attention mechanism to solve the difference of contained emotion information in different modes and different images. Firstly, the middle representation of each modal is fed to the local attention network and generates an emotion score for each image, and features of each modal will be aggregated according to their emotion scores. Secondly, features of each modal are fed to the global attention network and generate an emotion score for each modal, and the score and feature of multiple modes will be aggregated and the final emotion representation of the video will be produced. The performance of the HAMF network is evaluated and it can achieve excellent results on our MHED dataset.

Although our HAMF method obtains a promising performance in human emotion recognition in the video, because of the sparseness of emotional expression in the video, most videos contribute little to emotional recognition. Video emotion recognition mainly depends on some key video frames or clips. In the next, we will focus on extract and study videos containing rich emotions.

## Figures and Tables

**Figure 1:** Illustration of our motivation.

**Figure 2:** Example frames of each emotion category from the MHED dataset. (a) Anger. (b) Disgust. (c) Fear. (d) Joy. (e) Sadness. (f) Surprise.

**Figure 3:** Hierarchical attention-based multimodal fusion network.

**Figure 4:** Samples with their emotion scores predicted by HAMF.

**Figure 5:** Emotional scores of different modes of samples in Figure 4.

**Table 1:** Distribution of gender and age of MEHD dataset.

Ages	The number of males	The number of females
20–30	2	2
30–40	2	2
40–50	2	2
50–60	2	2

**Table 2:** The number of videos per category in MHED dataset.

Category	Anger	Disgust	Fear	Joy	Sadness	Surprise	Total
Number	145	157	137	220	226	181	1066
Average duration(s)	14.62	8.98	16.57	12.43	27.60	12.11	15.76

**Table 3:** Accuracy of emotion recognition of different modals.

Convolution layers	Face features accuracy (%)	Scene features accuracy (%)	Image features accuracy (%)
*L*1	55.14	44.39	46.03
*L2*	57.94	44.62	42.99
*L*3	54.67	43.92	44.62

**Table 4:** Accuracy of emotion recognition of global attention network.

Fully connected layers	Accuracy (%)
*G*1	62.15
*G*2	63.08
*G*3	61.92

**Table 5:** Accuracy of emotion recognition of different modals on Ekman and VideoEmotion-8 datasets.

Ekman			VideoEmotion-8		
Convolution layers	Event (%)	Object (%)	Scene (%)	Event (%)	Object (%)	Scene (%)
No attention	42.45	36.43	40.95	48.10	46.45	46.33
*L*1	44.14	41.42	44.41	51.34	49.88	49.14
*L*2	45.78	41.14	44.69	53.18	49.63	49.39
*L*3	45.23	40.33	43.60	52.81	48.90	49.02

**Table 6:** Accuracy of emotion recognition of global attention on Ekman and VideoEmotion-8 datasets.

Fully connected layers	Ekman (%)	VideoEmotion-8 (%)
No attention fusion	47.9	49.3
*G*1	56.68	52.69
*G*2	57.7	53.13
*G*3	55.31	51.71

**Table 7:** Performance evaluation of attention mechanism.

Methods	No attention accuracy (%)	Attention accuracy (%)
Face	51.87	57.94
Scene	44.16	45.09
Images	43.92	46.03
Fusion	60.05	63.08

**Table 8:** Top-1 accuracy (%) comparing state-of-the-art methods on MHED.

Method	Result (%)
Quality-aware network [12]	46.03
Barros et al. [22]	53.73
Chen et al. [10]	55.60
Kosti et al. [9]	56.07
Attention clusters [13]	59.81
Ours	63.08

**Table 9:** Top-1 accuracy (%) comparing state-of-the-art methods on Ekman-6 and VideoEmotion-8.

Method	Ekman (%)	VideoEmotion-8 (%)
Emotion in context [10]	51.8	50.6
Xu et al. [33]	50.4	46.7
Kernelized feature [26]	54.4	49.7
Concept selection [27]	54.40	50.82
Graph-based network [36]	55.01	51.77
CAAN [37]	56.23	52.5
Ours	57.7	53.13

## Data Availability

Ekman-6 and VideoEmotion-8 are two public datasets. The MHED dataset can be obtained from the corresponding author upon request.
